The article "On the Heterogeneity of Existing Repositories of Movements Intended for the Evaluation of Fall Detection Systems" was published in 2020. Journal: J Healthc Eng.

# On the Heterogeneity of Existing Repositories of Movements Intended for the Evaluation of Fall Detection Systems

**DOI:** 10.1155/2020/6622285

**Published:** 2020-11-30

**Authors:** Eduardo Casilari, José A. Santoyo-Ramón, José M. Cano-García

**Affiliations:** Departamento de Tecnología Electrónica, Universidad de Málaga, ETSI Telecomunicación, 29071 Málaga, Spain

## Abstract

Due to the serious impact of falls on the autonomy and health of older people, the investigation of wearable alerting systems for the automatic detection of falls has gained considerable scientific interest in the field of body telemonitoring with wireless sensors. Because of the difficulties of systematically validating these systems in a real application scenario, Fall Detection Systems (FDSs) are typically evaluated by studying their response to datasets containing inertial sensor measurements captured during the execution of labelled nonfall and fall movements. In this context, during the last decade, numerous publicly accessible databases have been released aiming at offering a common benchmarking tool for the validation of the new proposals on FDSs. This work offers a comparative and updated analysis of these existing repositories. For this purpose, the samples contained in the datasets are characterized by different statistics that model diverse aspects of the mobility of the human body in the time interval where the greatest change in the acceleration module is identified. By using one-way analysis of variance (ANOVA) on the series of these features, the comparison shows the significant differences detected between the datasets, even when comparing activities that require a similar degree of physical effort. This heterogeneity, which may result from the great variability of the sensors, experimental users, and testbeds employed to generate the datasets, is relevant because it casts doubt on the validity of the conclusions of many studies on FDSs, since most of the proposals in the literature are only evaluated using a single database.

## 1. Introduction

Falls, in particular falls among elderly, are a major social concern in current societies. The World Health Organization has reported that 646,000 persons die from falls each year worldwide, so they represent the second cause of unintentional injury deaths after car accidents [1]. In this respect, it has been shown that a rapid response after a fall can lower the risk of hospitalization by 26% and the death rate by 80% [2]. As a consequence, during the past decade, great research efforts have been devoted to the development of efficient and low-cost technologies for automatic Fall Detection Systems (FDSs).

Falls are generically and ambiguously defined as a loss of balance or accident that causes an individual to rest involuntarily on the ground or other lower level [3]. Most unintentional falls can be easily distinguished from other movements by human visual inspection. However, this task is not so evident when it is carried out by an automatic system. Accordingly, the problem of fall detection has been addressed through different approaches, which can be clustered into two great generic strategies: context-aware and wearable systems. Under the first strategy, an FDS can be deployed by placing video cameras and other ambient sensors, such as pressure sensors and microphones, in the vicinity of the user to be monitored. However, in most practical cases, the mobility of the patients can be tracked in a more adaptive and cost-effective way by employing lightweight sensors that can be directly transported on the clothes or as another garment or a piece of jewelry (e.g., as a pendant). The decreasing costs and widespread popularity of electronic wearables and especially those intended for sporting activities have fostered the adoption of this type of transportable solutions to investigate and implement FDSs. Under a wearable FDS, a detection algorithm is permanently in charge of analyzing the signals captured by the sensors worn by the user to identify any anomalous mobility pattern that can be linked to the occurrence of a fall. As soon as a fall is presumed, an alerting message (phone call and SMS) to a remote monitoring point (medical premises and patients' relative) will be forwarded by the FDS. In the vast majority of wearable architectures, the detection decision is based on the measurements provided by an accelerometer and, in some cases, a gyroscope (integrated in the same Inertial Measurement Unit, IMU), which are attached to a certain part of the user's body.

The general goal of an FDS is to simultaneously minimize both the number of falls that remain unnoticed and the generation of false alarms, that is to say, conventional movements or Activities of Daily Living (ADLs) that are misinterpreted as falls. A crucial element in the investigation of a wearable FDS is the procedure by which the detection algorithm will be methodically evaluated to check its actual capacity to discriminate ADLs from falls.

In almost all works existing in the related literature, FDSs are tested against a set of labelled movements that include both ADLs and falls. In order to repeat the analysis by changing the detection techniques and the parameterization of the algorithms, the movements are previously prerecorded in files that contain the corresponding timestamp and measurements gathered by the inertial sensors. The quality and representativeness of the employed dataset of movements are a key aspect to assess the validity of the evaluation. In this regard, it has been estimated that it is necessary to record between 70,000 and 100,000 days to collect about 100 actual falls by continuously monitoring persons aged over 65 [4]. Owing to the obvious practical difficulties of monitoring actual falls experienced by elderly people, the general procedure followed by the literature to evaluate a fall detection algorithm is using datasets of activity traces thatare intentionally created by experimental users. For this purpose, the participants in the experiments normally execute a series of predetermined movements while they transport the corresponding wearable sensors in one or several positions of their bodies. These movements typically incorporate different types of conventional ADLs (sitting, climbing stairs, picking up objects from the floor, etc.) and falls, which are mimicked taking into account different aspects, such as the direction (lateral and backwards) or the cause of the fall (slipping, stumbling, and tripping).

In almost all initial studies on FDSs, a group of volunteers were recruited to generate a specific dataset which was employed for the evaluation of the proposed architecture. These datasets were rarely released by the authors to enable their use by other researchers to validate new algorithms. To tackle this lack of a benchmarking framework, a nonnegligible number of datasets have recently been produced and made publicly available on the Web to cross compare FDSs with a common reference.

The use of normally young and healthy volunteers that emulate falling in a systematic way in a ‘controlled' scenario, as surrogates for actual falls of older persons, is still a controversial issue in the field of FDSs. By tracking during six months two groups of persons totaling 16 older people, Kangas et al. conducted a study aiming at comparing the dynamics of real-life falls of older people with those simulated by middle-aged volunteers [5]. From the results, the authors concluded that the features of the acceleration data captured during accidentals falls follow a similar pattern to those measured from emulated falls, although some significant differences were detected (for example, in the timing of the different phases of the falls or in the acceleration magnitude measured during the impact against the floor). In a similar study [6], Klenk et al. compared the actual backward falls suffered by four elderly people to those mimicked by 18 young individuals. Results seem to indicate that the ‘compensation' strategies to avoid the damages of the impact followed by the subject during the unintentional falls introduce relevant differences (e.g., jerkier movements with higher changes in the acceleration) with respect to the case of the emulated falls.

Besides, Bagalà et al. [7] have shown that the efficacy of certain algorithms successfully tested against datasets of emulated falls may notably decrease when they are evaluated with traces captured in a real scenario. In other works, such as that by Sucerquia et al., the ability of the proposed FDS to avoid false alarms is evaluated by monitoring elderly people that transport the wearable detection system during their daily routines. In these cases, the sensitivity of the detector cannot be computed unless a real fall occurs during the monitoring period. A similar strategy is described by Aziz et al. in [8]. These authors report that the number of false alarms of an FDS, which is based on a Support Vector Machine classifier, deteriorates when it is employed by a community of 19 older adults. In this scenario, 2 out of 10 actual falls suffered by the participants were not identified by the system.

In any case, these studies are based on the analysis of a very small number of real falls. The fact is that, to the best of our knowledge, the repository provided by the FARSEEING European project [9] is the only dataset that provides inertial measurements of real-world falls of elderly patients although again the number of samples that are publicly available, only 22, is quite limited. Thus, this work mainly focuses on those datasets grounded on emulated falls and ADLs (although in some cases, ADLs were captured not by an execution of predetermined activities on a laboratory but by monitoring the participants during their daily routines).

On the other hand, although the use of public and well-known datasets is gaining an increasing acceptance in the literature, most studies base their validation on the use of just one or, at most, two repositories. So, a question arises about the correctness of extrapolating the results obtained with a particular dataset when another repository is considered.

The goal of this study is to recap and compare the characteristics of the existing public repositories of inertial measurements intended for the assessment of FDSs.

The paper is organized as follows.  Section 2 revises the available datasets, synopsizing their basic properties and the testbeds (employed sensors, characteristics of the experimental users, and typology of the movements) which were deployed to generate the data. The section also describes the criteria to select the datasets to be compared.  Section 3 presents the statistical features employed to characterize the mobility of the traces of the datasets, while Section 4 compares the datasets by showing the results of the analysis of variance (ANOVA) of these characteristics. The main conclusions are summarized in Section 5.

## 2. Revision and Selection of Public Datasets

As aforementioned, a key problem for the development of an automatic fall detection architecture is the need of trustworthy repositories that can be employed to thoroughly evaluate the accuracy of the detection decisions, i.e., the capacity of the system to correctly identify ADLs and falls by simultaneously avoiding false alarms and undetected falls.

Table 1 presents a comprehensive list of the authors, references, institutions, and year of publication of the existing datasets intended for the study of wearable systems. All these datasets comprise the measurements collected by the inertial sensors worn by the selected volunteers during their daily life or while performing a preconfigured set of movements in a controlled testbed. In this revision we do not include those available databases of inertial measurements (such as those presented in [10] or [11]) that are envisioned for other types of HAR (Human Activity Recognition) systems but do not incorporate falls among the represented activities .

In the case of Context-Aware Systems (CAS), different research groups have also published datasets containing the measurements captured by fixed video camera, motion and depth sensors (such as Kinect), and/or other ambient sensors (vibration detectors, pressure, infrared, and Doppler sensors, and near-field imaging systems), while a set of volunteers emulate falls and ADLs in a predefined testbed. Among these databases, we can mention the following: CIRL Fall Recognition [12], Le2i FDD [13], SDUFall [14], EDF&OCCU [15], eHomeSeniors [16], Multiple Camera Fall [17] KUL High-Quality Fall Simulation [18], UTA [19], FUKinect-Fall [20], or MEBIOMEC [21] datasets, as well as the infrared video clips described by Mastoraky and Makris in [22] or those sequences provided by Adhikari et al. in [23]. These datasets are out of the scope of this paper although we do consider those databases, such as UR Fall or UP Fall, which were conceived to test hybrid CAS-type and wearable FDSs, i.e., systems that make their detection decision from the joint analysis of video images (and/or magnitudes collected by environmental sensors) and measurements from inertial sensors transported by the users.

The number of samples, the considered typologies of the emulated ADLs and falls, and the duration of the traces (i.e., the duration of the recorded movements), as well as the basic characteristics of the participants (number, gender, weight, and age range) of each dataset, are enumerated in Table 2.

Table 2 illustrates the great heterogeneity of criteria used to define the experimental framework where the samples were captured, both with regard to the selection of the test subjects and the number and type of simulated movements. In some repositories, such as tFall, the ADLs were not emulated (scheduled and executed in a laboratory) but obtained by tracking the real-life movements of the subjects during a certain period of time. As expected, in most cases, the movements were exclusively carried out by volunteers under the age of 60. In the few testbeds in which older subjects participated, almost none of the older participants simulated any fall, so their samples are limited to examples of ADLs.

Table 3 summarizes, in turn, the type and basic properties (sampling rate and range) of the sensors employed to generate the repositories. The table also indicates the corporal position on which the inertial sensors were located or attached during the experiments. As it can be observed from the table, although there are cases where up to seven sensing positions have been considered, most datasets include just a single measuring point. In all cases, the sensor embeds, at least, an accelerometer and, less often, a gyroscope, a magnetometer, and/or an orientation sensor. In any case, the table shows the variability of the characteristics of the sensors (e.g., with sampling rates ranging from 10 to 200 Hz) and the body location considered to collect the measurements in the different testbeds again.

In the recent literature about FDSs, the use of some of these public datasets as benchmarking tools is becoming more and more common. However, in most studies, just one or, at most, two repositories are utilized to evaluate the effectiveness of the proposed detection algorithm. Khojasteh et al. [24] employed four datasets, although two of them (DaLiac [25] and Epilepsy [26] databases) do not encompass falls, which only allows assessing the capability of the system to avoid misinterpreting ADLs as falls. As a consequence, the conclusions of most works are mainly based on the results obtained when the proposed system is tested against a very particular set of samples.

Given the huge diversity of the experimental setups in which the datasets were generated, it is legitimate to question whether the conclusions achieved with a certain repository can be extrapolated to scenarios with a different typology of subjects, movements (simulated or not), or to a different parameterization of the inertial sensors.

In this context, Medrano et al. utilized three repositories (tFall, DLR, and MobiFall) in [27] to show that the effectiveness of an FDS based on a supervised machine learning strategy remarkably diminishes when the discrimination algorithms are tested against a database different from that utilized for training. In a more recent work [28], we concluded that even when the algorithm is trained and tested with traces of the same datasets and users, the quality metrics of the classification process may differ notably. In particular, we analyzed the performance of a deep learning classifier (a convolutional neural network) when it is individually trained and evaluated as a fall detector with 14 of the repositories presented in Table 1. Results clearly indicated that the performance dramatically varies depending on the dataset to which the detector is applied.

In the following sections, we thoroughly analyze the statistical properties of a representative number of these datasets to get a deeper understanding of the existing divergences between these repositories.

### 2.1. Election of the Compared Datasets

In order to compare the properties of the signals provided by different repositories on equal terms, we only select those datasets that contain inertial measurements captured on the same position. In particular, in a first analysis, we focus on those traces collected on the waist as several studies [53–57] have shown that this is one of the most adequate positions to place an inertial sensor aimed at characterizing the general dynamics of the body. This election benefits from the fact that the waist is near the center of mass of the human body in a standing posture. When compared to other placements such as a limb or the chest, the waist also provides better ergonomics as it may enable the user to transport the wearable sensor almost in a seamless way (e.g., attached to a belt).

To ensure that the analysis is performed with a minimum number of samples, we only take into account those datasets with, at least, 300 samples. Consequently, we discard UR, FARSEEING, LDPA, and TST datasets, although they include traces captured with the sensor located on the waist. For a similar reason, we exclude the SMotion dataset [45], which is actually aimed at assessing fall risk and not fall detection systems, as it only contains 5 falls.

Finally, the Graz UT OL dataset is also discarded because of the small range of the employed accelerometer (±2g), which can prevent a proper representation of the acceleration peaks caused by falls (typically exceeding 4-5g).

## 3. Selection of the Characteristics for the Analysis

As in most works in the literature, the study will be based on the signals collected by the triaxial accelerometers (*A*_*X*_[*i*], *A*_*Y*_[*i*], *A*_*Z*_[*i*] for the *i*-th measurement), which are provided by the datasets. Future studies should contemplate the analysis of the signals collected by the gyroscope and, secondarily, the magnetometer. Nevertheless, it is still under discussion that the information provided by the gyroscope may significantly improve the success rate of methods merely based on the accelerometry signals (see [58] for a revision of this issue).

During the free-fall period before the impact, a collapse typically prompts a sudden drop of the acceleration components, which is interrupted by a sharp peak of the acceleration magnitude (sometimes followed by several secondary peaks) produced by the collision against the floor [59]. Therefore, to define a common basis to compare the traces, which present a wide variety of lengths, we focus on the interval of every measurement sequence where the highest difference between the “valleys” (decays) and peaks of the acceleration components is detected. Once this analysis interval is extracted, the rest of the trace is ignored. For this purpose, we set up a sliding observation window of duration *t*_*W*_ = 0.5 s, consisting of *N*_*W*_ samples:

(1) $$\begin{array}{c} N_{W}=t_{W}\cdot f_{s}, \end{array}$$

where *fs* indicates the sampling rate of the sensors.

To find the analysis interval within each trace, we follow the procedure presented in [60]. Thus, for each possible observation window within the sequences, we calculate the magnitude of the maximum variation of the acceleration components (*A*_*w*_diff__[*m*]) as

(2) $$\begin{array}{c} A_{w_{\text{diff}}}\left[m\right]=\sqrt{{\left(A_{X_{\text{max}}}\left[m\right]-A_{X\text{min}}\left[m\right]\right)}^{2}+{\left(A_{Y_{\text{max}}}\left[m\right]-A_{Y\text{min}}\left[m\right]\right)}^{2}+{\left(A_{Z_{\text{max}}}\left[m\right]-A_{Z\text{min}}\left[m\right]\right)}^{2}\;}, \end{array}$$

where *A*_*X*_max__[*m*], *A*_*Y*_max__[*m*], and *A*_*Z*_max__[*m*]*d*esignate the maximum values of the components measured by the accelerometer in the *x*-, *y*- and *z-*axis, respectively, in the *m*-th sliding observation interval. Thus, for the *x*-axis, we have

(3) $$\begin{array}{c} A_{X_{\text{max}}}\left[m\right]=\text{max}\left(A_{X}\left[i\right]\right),\;\forall i\in \left[m,m+N_{W}-1\right]. \end{array}$$

The analysis or observation interval will correspond to the subset of consecutive samples [*k*_*o*_, *k*_*o*_+*N*_*W*_ − 1] where the maximum *A*_*w*_diff(max)__ of *A*_*w*_diff__[*m*] is located:

(4) $$\begin{array}{c} A_{w_{\text{diff}\left(\text{max}\right)}}=A_{w_{\text{diff}}}\left[k_{o}\right]=\text{max}\left(A_{w_{\text{diff}}}\left[m\right]\right),\\ \;\forall m\in \left.\left[1,N-N_{W}+1\right]\right), \end{array}$$

where *k*_*o*_ is the index of the first sample of the analysis interval while *N* denotes cardinality (number of samples for each axis) of the trace.

In order to compare the different datasets, we extract the acceleration components of the signals during the analysis interval to compute the following twelve statistical features for all the traces. 

All these features have been regularly employed by the related literature on FDSs and human activity recognition systems (see, for example, the FDS described in [37, 43, 54, 61–72] or the comprehensive analyses presented by Vallabh in [73] or by Xi in [74]).

1. The mean Signal Magnitude Vector (*µ*_**SMV**_), which gives an idea of the average mobility experienced by the body during the analysis interval. This mean can be calculated as

(5) $$\begin{array}{c} {µ}_{\text{SMV}}=\frac{1}{N_{W}}\cdot \sum_{i=k_{o}}^{k_{o}+N_{W}-1}\text{SMV}\left[i\right], \end{array}$$

  where SMV[*i*] represents the Signal Magnitude Vector (SMV) of the acceleration for the *i*-th sample:

(6) $$\begin{array}{c} \text{SMV}\left[i\right]=\sqrt{{\left(A_{X}\left[i\right]\right)}^{2}+{\left(A_{Y}\left[i\right]\right)}^{2}+{\left(A_{Z}\left[i\right]\right)}^{2}}. \end{array}$$

(2) The standard deviation (*σ*_**SMV**_) of SMV[*i*], which describes the variability of the acceleration during the observation window:

(7) $$\begin{array}{c} \sigma_{\text{SMV}}=\sqrt{\frac{1}{N_{W}}\cdot \sum_{i=k_{o}}^{k_{o}+N_{W}-1}{\left(\text{SMV}\left[i\right]-{µ}_{\text{SMV}}\right)}^{2}\;}. \end{array}$$

(3) The mean absolute difference (*μ*_**SMV**_**diff**__) between two consecutive samples of the acceleration module, which is estimated as

(8) $$\begin{array}{c} \mu_{{\text{SMV}}_{\text{diff}}}=\frac{1}{N_{W}}\cdot \sum_{i=k_{o}}^{k_{o}+N_{W}-1}\left|\text{SMV}\left[i+1\right]-\text{SMV}\left[i\right]\right|. \end{array}$$

  This parameter is useful as it informs about the brusque fluctuations of the acceleration during a fall [75].
(4) The mean rotation angle (*µ*_*θ*_) may help to detect the changes of the body orientation of the body caused by a fall [75]. This angle is computable as

(9) $$\begin{array}{c} {µ}_{\theta }=\frac{1}{N_{W}}\cdot \sum_{i=k_{o}}^{k_{o}+N_{W}-1}\left({\text{cos}}^{-1}\left[\frac{A_{X}\left[i\right]\cdot A_{X}\left[i+1\right]+A_{Y}\left[i\right]\cdot A_{Y}\left[i+1\right]+A_{Z}\left[i\right]\cdot A_{Z}\left[i+1\right]\;}{\text{SMV}\left[i\right]\cdot \text{SMV}\left[i+1\right]}\right]\right). \end{array}$$

(5) The acceleration component in the direction perpendicular to the floor plane is strongly determined by the gravity. Thus, the tilt of the body provoked by the falls usually triggers a noteworthy alteration of the acceleration components that are parallel to the floor plane when the individual remains static in an upright posture. To characterize the alteration of the body position with respect to the standing position, we also compute the **mean magnitude (***µ*_**Ap**_**)** of the vector formed by these two acceleration components:
  (10) $$\begin{array}{c} {µ}_{Ap}=\frac{1}{N_{W}}\cdot \sum_{i=k_{o}}^{k_{o}+N_{W}-1}\sqrt{{\left(A_{H1}\left[i\right]\right)}^{2}+{\left(A_{H2}\left[i\right]\right)}^{2}}, \end{array}$$
where the pair (*A*_*H*1_[*i*],*A*_*H*2_[*i*]) of acceleration components may alternatively represent (*A*_*X*_[*i*],*A*_*Y*_[*i*]) (*A*_*X*_[*i*],*A*_*Z*_[*i*]) or (*A*_*Y*_[*i*],*A*_*Z*_[*i*]) depending on the placement and orientation of the accelerometer in each dataset.
(6) The aforementioned value of **A**_**w**_**diff**(*max*)__, which gives an insight of the range of the variability of the three acceleration components.
(7) The peak or maximum (**SMV**_**max**_)of the SMV, as a key element to describe the violence of the impact against the floor:
  (11) $$\begin{array}{c} {\text{SMV}}_{\text{max}}=\text{max}\left(\text{SMV}\left[i\right]\right),\;\forall i\in \left[k_{o},k_{o}+N_{W}-1\right]. \end{array}$$
(8) The “valley” or minimum (**SMV**_**min**_) of the SMV to characterize the phase of free-fall:
  (12) $$\begin{array}{c} SMV_{min}=\text{min}\left(\text{SMV}\left[i\right]\right),\;\forall i\in \left[k_{o},k_{o}+N_{W}-1\right]. \end{array}$$
(9) The skewness of SMV[*i*] (*γ*_**SMV**_), which describes the symmetry of the distribution of the acceleration:
  (13) $$\begin{array}{c} \gamma_{\text{SMV}}=\frac{1}{\sigma_{\text{SMV}}^{3}\cdot N_{W}}\cdot \sum_{i=k_{o}}^{k_{o}+N_{W}-1}{\left(\text{SMV}\left[i\right]-{µ}_{\text{SMV}}\right)}^{3}. \end{array}$$
(10) The Signal Magnitude Area (**SMA**) [43]. This parameter, which is an extended feature used to evaluate the physical activity, can be estimated as
  (14) $$\begin{array}{c} \text{SMA}=\frac{1}{N_{W}}\cdot \sum_{i=k_{o}}^{k_{o}+N_{W}-1}\left(\left|A_{X}\left[i\right]\;\right|+\left|A_{Y}\left[i\right],\;\right|+\left|A_{Z}\left[i\right]\;\right|\right). \end{array}$$
(11) Energy (***E***). Since falls are associated to rapid and energetic movements, we also consider the sum of the energy (*E*) estimated in the three axes during the observation interval [72]:
  (15) $$\begin{array}{c} E=\frac{1}{N_{W}}\cdot \left(\sum_{i=0}^{N_{W}-1}{\left|{\text{FFT}}_{X}\left[i\right]\right|}^{2}+\sum_{i=0}^{N_{W}-1}{\left|{\text{FFT}}_{\text{Y}}\left[i\right]\right|}^{2}+\sum_{i=0}^{N_{W}-1}{\left|{\text{FFT}}_{Z}\left[i\right]\right|}^{2}\right), \end{array}$$
where FFT_*X*_[*i*], FFT_*Y*_[*i*], and FFT_*Y*_[*i*], respectively, indicate the Discrete Fourier Transform of the acceleration components *A*_*X*_[*i*],*A*_*Y*_[*i*], and *A*_*Z*_[*i*] in the analysis interval, straightforwardly computable (for the *x*-axis) as
  (16) $$\begin{array}{c} {\text{FFT}}_{X}\left[i\right]=\sum_{m=0}^{N_{W}-1}A_{X}\left[k_{o}+m\right]\;\cdot e^{-j2\pi \left(im/N_{W}\right)},\\ \;\text{for }i=0,1,\ldots ,N_{W}-1. \end{array}$$
(12) Mean of the autocorrelation function (*μ*_**R**_) of the acceleration magnitude captured during the observation interval:
  (17) $$\begin{array}{c} \mu_{R}=\frac{1}{N_{W}}\cdot \sum_{l=0}^{N_{W}-1}R\left[m\right], \end{array}$$

where *R*[*m*] represents the *m*-th lag value in the series of the normalized autocorrelation coefficients of SMV[*i*]:

(18) $$\begin{array}{c} R\left[m\right]=\frac{1}{\sigma_{\text{SMV}}^{2}\cdot N_{W}}\cdot \left(\sum_{i=k_{o}}^{k_{o}+N_{W}-m-1}\left(\text{SMV}\left[i\right]-{µ}_{\text{SMV}}\right)\left(\text{SMV}\left[i+M\right]-{µ}_{\text{SMV}}\right)\right),\;\text{for }m=0,\;1,\;\ldots ,N_{W}-1. \end{array}$$

This feature *μ*_*R*_ is taken into account as long as the acceleration during a conventional activity normally exhibits a certain degree of self-correlation that could be impacted by the unexpected movements caused by a fall.

## 4. Comparison and Discussion of the Datasets

For an initial comparison of the statistical features of the different datasets, we utilize boxplots (or box-and-whisker plots), an extended and intuitive visual tool, to display the data distribution in a standardized manner.

Figures 1–12 show the boxplots of the twelve statistics when they are separately calculated for the ADLs and the fall movements of the seven datasets under study. In the graphs, for each dataset and type of activity (ADL/fall), the median of the corresponding statistic is denoted by the central line in each box while the 25th and 75th percentiles are indicated by the lower and upper limits of the box. The dotted lines or “whiskers” represent an interval over and under the box of 1.5 IQR (the height of the box or Interquartile range between the 25th and 75th percentiles). All the data outside these margins (box and whiskers) are considered to be outliers and marked as red crosses in the figures.

The graphs show the high inter- and intravariability of the statistics of the traces. As it refers to the intravariability, within each repository, the analysis identifies a wide IQR interval and a high number of outliers for almost all the characteristics, in particular for the ADLs. Similarly, when the boxplots of the different databases are compared, a huge heterogeneity is also present.

This intravariability among datasets is also noticeable (both for ADLs and falls) even in the case of a basic feature, such as the mean acceleration magnitude during the observation window (which is assumed to be linked to the period of greatest alteration in the body acceleration). For all the considered statistics and for both ADLs and falls, we can observe several pairs of datasets where the IQR intervals (which concentrate 50% of the samples) do not even overlap, i.e., the 25% quartile of the corresponding feature of a certain dataset exhibits a higher value than that of the 75% quartile for the same feature of a different dataset. In addition, the magnitude of the IQR interval strongly differs from one repository to another. In some cases, the estimated mean of certain statistics in one dataset is several times higher when compared to others. This is more visible for those characteristics associated with the loss of verticality: the mean rotation angle (*µ*_*θ*_) and the mean magnitude of the acceleration components (*µ*_*Ap*_) perpendicular to the vertical plane while standing.

The statistical significance of these divergences among the repositories can be systematically confirmed by an ANOVA (Analysis of variance) test. Figures 13 and 14 depict the post hoc multiple comparison of the estimated means of the twelve features based on the results achieved by a one-way (or single-factor) ANOVA. In the bars of the figure, the circular marks indicate the mean whereas the corresponding comparison interval for a 95% confidence level is represented by the line extending out from the symbol. The group means are considered to be significantly different if the intervals determined by the lines are disjoint.

Each subgraph in these two figures shows, in red, those datasets that have a characteristic with a significantly different mean than that of the fall or ADL movements of another dataset (marked in blue), which is taken as a reference by way of an example. As can be seen in the figure, there are very few cross comparisons, indicated in grey, in which the null hypothesis is not rejected as the differences between the means of the characteristics are not significantly relevant.

This inconsistency in the characterization of the different datasets is also appreciated if we consider other duration of the time observation window in which the maximum variation of the acceleration components is detected. Figures 15 and 16 present the analysis of variance when it is applied to the features computed for two different observation intervals (0.5 s and 1 s, respectively). For the sake of simplicity, the graphs only show the six first characteristics although a similar disparity can be found if the other six features were shown.

### 4.1. Comparison of the Different Types of ADLs

The differences analyzed in the previous section could be partly justified by the fact that the terms ‘ADL' and ‘falls' may hide a huge variety of different movements. This is particularly true for the groups labelled as ADLs, as they can encompass activities ranging from those that require almost no effort, such as standing, to those that are much more physically demanding (such as running). In spite of this evident heterogeneity, the authors of the datasets normally select the typology of the ADLs to be emulated by the volunteers without previously discussing the degree of mobility that the selected activities actually require.

In order to minimize the effects of this heterogeneity in the ADLs, we propose to individualize the previous ANOVA study taking into account the nature (physical effort) of the ADLs. For this purpose, as we also suggested in [76], we split the ADLs of each repository into three generic subcategories: basic ordinary movements (such as getting up, sitting, standing, and lying down), standard routines that entail some physical effort or a higher degree of mobility or leaning of the body (walking, climbing up and down stairs, picking an object from the floor, and tying shoe laces), and finally, sporting activities (running, jogging, jumping, and hopping).

By taking into account this taxonomy, Table 4 displays and catalogues the different types of ADLs and falls contained in the seven datasets under analysis. The table shows that each subcategory in each dataset is basically represented by the same three or four types of common movements. Thus, a certain homogeneity could be presumed. In two of the datasets (DOFDA and IMUFD), there are no sporting activities. As an extra type of ‘nonfall' movements, the table also indicates which repository includes the emulation of near falls, that is to say, missteps, stumbles, trips, or any other type of accidental movements that involve a loss of balance but do not result in a fall.

The individualized ANOVA analyses of the series of the six statistical features of the datasets are depicted in Figures 17 and 18 (for basic movements), Figures 19 and 20 (for standard movements), and Figures 21 and 22 (for sporting movements).

Despite the categorization and clustering of the traces, the graphs again reveal the great variability of the datasets when they are compared to each other. For all three movement types and for all metrics, the mean of the six statistical features of each dataset is significantly different from that calculated for, at least, two other datasets. Figures evince that in a nonnegligible combination of cases (some of which are highlighted in blue in the graphs), the null hypothesis can be rejected for the comparison of a certain mean of a particular dataset with the mean of the same metric of the rest of datasets. For example, five out of the six contemplated features in the basic movements of the UMAFall repository present a mean value significantly different to those of all the other datasets. A similar behavior is detected in other repositories and types of movements (e.g., the sporting activities in the UP dataset).

A similar conclusion can be reached by analyzing the near-fall movements existing in two datasets (IMUFD and Erciyes). Figures 23 and 24 confirm that the six statistics with which these movements have been characterized present mean values that significantly differ for the two repositories.

### 4.2. Comparison for the Same Type of Movement: Walking

The disparity in the statistical characterization of the traces is confirmed even when the same type of movement is considered as the basis for comparing the datasets. Figures 25 and 26 depict the results obtained when the ANOVA is exclusively applied to those movement samples (measured on the waist) labelled as “walking”. We select this ADL due to its importance in real-life scenarios of FDSs as it is the movement that normally precedes falls and because it is present in the seven datasets (DLR, DOFDA, Erciyes, IMUFD, SisFall, UMAFall, and UP-Fall) that employ a sensor on the waist. As it can be appreciated from the figures, even for a common physical activity as walking, the characteristics show noteworthy discrepancies among the datasets. Figures show that there are only three characteristics (*σ*_SMV_, *A*_*ω*_diff(max)__, and SMV_max_) for which the null hypothesis cannot be rejected as long as no dataset exhibits a mean that can be considered significantly different from those computed for other databases. For some characteristics (for example, note the absence of overlapping intervals in the graphs corresponding to *μ*_*θ*_ or *μ*_*R*_) the post hoc tests show that all or almost all datasets are significantly different.

### 4.3. Results for the Measurements on the Wrist

To corroborate the previous results, we apply the previous analysis to the datasets containing measurements captured on a completely different body position: the wrist. In spite of the particular (and independent) mobility of the wrist, this position has been selected in a significant number of studies on FDSs as the position to locate the detection sensor. The wrist offers to the user better ergonomics than other typical placements as humans are already habituated to wear watches. Moreover, commercial smartwatches (which are natively provided with inertial measurement units) can be employed to deploy the FDS without obliging the user to transport any supplementary device. In some articles that consider systems with more than one sensing mote, the wrist-sensor can be used as a backup node to confirm the detection decision taken from the measurements obtained on another body area.

To extend the study to the wrist-based measurements, we repeat the selection process described in Section 3 and select only those datasets that employed a sensor on that position in the datasets (see Table 3). Thus, six datasets were selected: Erciyes, UP-Fall, and UMAFall (already utilized in the previous analysis of the traces obtained from the waist), as well as CMDFall, SmartFall, and Smartwatch datasets.

The results of the ANOVA analysis of the series of the twelve statistical features of these six datasets (when an observation window is contemplated) are represented in Figures 27 and 28 (for ADLs) and Figures 29 and 30 (for the fall movements).

As expected, the graphs show even a higher disparity between the datasets than those obtained on the waist.

The way in which the volunteers are instructed to execute the ADLs and falls may particularly determine the position and movements of the hands during the activities. Thus, the measured dynamics may be extremely dependent on the testbed, which reduces the suitability of the traces for being extrapolated to other scenarios.

### 4.4. Discussion

This heterogeneity of the repositories can be motivated by very different factors, which we could group as follows:

- Technological factors: inertial sensor problems and limitations (biases, calibration issues, and range) can affect the measurements
- Ergonomic factors: although we have compared datasets where the measurements were taken in a similar body area (the waist), measurements could be altered by the exact position of the sensor, the discomfort that the sensing device can cause in the user (which could influence the naturalness of the movements), or the firmness with which the device is adjusted to the body
- Factors determined by the design of the testbed: the variability of the datasets could be clearly justified not only by the intrinsic variability (in number and types) of the performed movements but also by the particularities of the physical setting in which the movements take place: the route of the subjects during the execution of each activity, the external elements (stairs, chairs, and beds) used in the routines, or the mechanisms used to cushion the impact of the falls (mattresses, elbow pads, and helmets)
- Human factors: finally, the data could be affected not only by the criteria for choosing the subjects (especially the age) but also by the particular training (or orders) that the volunteers receive to carry out the activities (in particular the falls)

## 5. Conclusions

This paper has presented a thorough study of the existing public repositories employed in the validation of Fall Detection Systems (FDS) based on wearables. The paper compares and summarizes the main basic characteristics of up to 25 available datasets used as benchmarking tools in the evaluation of FDSs.

Due to the difficulties of obtaining inertial measurements of actual falls, all these databases (except one) were created by groups of volunteers that executed a predetermined set of ADLs (Activities of Daily Living) and mimicked falls in a controlled lab-type environment. In this regard, most works in the literature evaluate their proposals by analyzing their behavior when they are applied to just one (or at most two) of these datasets. In order to indirectly assess the validity of testing a certain FDS with a single dataset, we have systematically compared the statistical characteristics of the series contained in seven of these repositories. The selection criterion of the analyzed datasets was founded on the election of a common position (waist) in which the sensor was located and on the cardinality of the measurement sets. In any case, by also analyzing the movements captured on the wrist, we also showed that conclusions could be extrapolated if other body locations with a higher degree of movement autonomy are considered.

The study, which was restricted to the accelerometry signals (as they are massively employed by the related literature on FDSs), defined and computed twelve statistical features to characterize different properties of the human mobility for each activity during the observation window (of fixed duration) in which the maximum variation of the acceleration magnitude is detected. The analysis was repeated with up to three different observation intervals without identifying a strong coherence in the characteristics obtained from the analysis of the different traces.

In particular, by means of an ANOVA analysis, we compared the means of the different statistics taking into account the nature (falls or ADLs) of the activity. This comparison was repeated after clustering the ADLs into three subcategories (basic, standard, and sporting activities) depending on the physical effort that they demand. In all cases, a significant difference of the means was found for almost all the datasets and features. Same conclusions were drawn even when a unique and simple type of standard movement (walking) was selected to compare the databases.

The divergence of the datasets could be justified by the complex interaction of a wide set of factors: the typology and number of activities (even for those in the same subcategory), the method to execute the programmed movements, the characteristics of the experimental subjects, the range, quality, and ergonomics of the sensors, the way in which the sensing device is fastened, and the elements employed to cushion the falls. In this sense, the study reveals an evident lack of consensus on the procedure followed to define the experimental testbeds in which the datasets are generated. For example, just one of the studied datasets includes (as nonlabelled ADLs) samples captured while monitoring the actual daily routines of the volunteers.

In any case, the heterogeneity of the datasets highlighted by this investigation calls into question the results of all those studies that test the FDS against a single repository. Thanks to the sophisticated methods currently used by the literature, normally based on machine learning or deep learning techniques, some studies have achieved quality metrics (sensitivity and specificity) in the recognition of ADLs and falls very close to 100%. However, these works do not normally evaluate the capability of these methods to extrapolate these positive results when using other datasets than those considered during the training and initial validation of the FDS.

With this in mind, we should not ignore either that the credibility of the research on FDS systems is still undermined by the lack of datasets with a representative number of real falls of older people (the target population of these emergency systems), which could be utilized to benchmark the detection methods in a more realistic scenario.

## Figures and Tables

**Figure 1:** Boxplots of the mean Signal Magnitude Vector (*μ*_SMV_) for the ADLs (left column) and falls. (a) ADLs. (b) Falls (right column) of all datasets.

**Figure 2:** Boxplots of the maximum variation of the standard deviation of the Signal Magnitude Vector (*σ*_SMV_) for the ADLs (left column) and falls (right column) of all datasets. (a) ADLs. (b) Falls.

**Figure 3:** Boxplots of the mean rotation angle (*µ*_*θ*_) for the ADLs (left column) and falls (right column) of all datasets. (a) ADLs. (b) Falls.

**Figure 4:** Boxplots of the mean absolute difference between consecutive samples (*μ*_SMV_diff__) for the ADLs (left column) and falls (right column) of all datasets. (a) ADLs. (b) Falls.

**Figure 5:** Boxplots of the mean module of the not perpendicular acceleration components (*µ*_*Ap*_) for the ADLs (left column) and falls (right column) of all datasets. (a) ADLs. (b) Falls.

**Figure 6:** Boxplots of the maximum variation of the acceleration components (*A*_*ω*_diff(max)__) for the ADLs (left column) and falls (right column) of all datasets. (a) ADLs. (b) Falls.

**Figure 7:** Boxplots of the maximum (SMV_max_) of the SMV for the ADLs (left column) and falls (right column) of all datasets. (a) ADLs. (b) Falls.

**Figure 8:** Boxplots of the minimum (SMV_min_) of the SMV for the ADLs (left column) and falls (right column) of all datasets. (a) ADLs. (b) Falls.

**Figure 9:** Boxplots of the skewness of *SMV* (*γ*_SMV_) for the ADLs (left column) and falls (right column) of all datasets. (a) ADLs. (b) Falls.

**Figure 10:** Boxplots of the Signal Magnitude Area (SMA) for the ADLs (left column) and falls (right column) of all datasets. (a) ADLs. (b) Falls.

**Figure 11:** Boxplots of the sum of the energy (E) estimated in the three axes for the ADLs (left column) and falls (right column) of all datasets. (a) ADLs. (b) Falls.

**Figure 12:** Boxplots of the mean of the autocorrelation function (*μ*_*R*_) for the ADLs (left column) and falls (right column) of all datasets. (a) ADLs. (b) Falls.

**Figure 13:** Multiple comparison test of the means of the following statistical characteristics of the datasets: (a) *μ*_**SMV**_. (b) *σ*_**SMV**_. (c) *μ*_*θ*_. (d) *μ*_**SMV**_(diff)__. (e) *μ*_**Ap**_. (f) **A**_*ω*_**diff**(**max**)__.

**Figure 14:** Multiple comparison test of the means of the following statistical characteristics of the datasets: (a) **SMV**_**max**_. (b) **SMV**_**min**_. (c) *γ*_**SMV**_. (d) SMA. (e) **E**. (f) *μ*_**R**_.

**Figure 15:** Multiple comparison test of the means of the statistical characteristics of the datasets: (a) *μ*_**SMV**_. (b) *σ*_**SMV**_. (c) *μ*_*θ*_. (d) *μ*_**SMV**_(**diff**)__. (e) *μ*_**Ap**_. (f) **A**_*ω*_**diff**(**max**)__. Observation window of 0.5 s.

**Figure 16:** Multiple comparison test of the means of the statistical characteristics of the datasets: (a) *μ*_**SMV**_. (b) *σ*_**SMV**_. (c) *μ*_*θ*_. (d) *μ*_**SMV**_(**diff**)__. (e) *μ*_**Ap**_. (f) **A**_*ω*_**diff**(**max**)__. Observation window of 2 s.

**Figure 17:** Multiple comparison test of the means of the statistical characteristics of the basic movements in the datasets: (a) *μ*_**SMV**_. (b) *σ*_**SMV**_. (c) *μ*_*θ*_. (d) *μ*_**SMV**_(**diff**)__. (e) *μ*_**Ap**_. (f) **A**_*ω*_**diff**(**max**)__. Basic movements.

**Figure 18:** Multiple comparison test of the means of the statistical characteristics of the basic movements in the datasets: (a) **SMV**_**max**_. (b) **SMV**_**min**_. (c) *γ*_**SMV**_. (d) SMA. (e) **E**. (f) *μ*_**R**_. Basic movements.

**Figure 19:** Multiple comparison test of the means of the statistical characteristics of the standard movements in the datasets: (a) *μ*_**SMV**_. (b) *σ*_**SMV**_. (c) *μ*_*θ*_. (d) *μ*_**SMV**_(**diff**)__. (e) *μ*_**Ap**_. (f) **A**_*ω*_**diff**(**max**)__. Standard movements.

**Figure 20:** Multiple comparison test of the means of the statistical characteristics of the standard movements in the datasets: (a) **SMV**_**max**_. (b) **SMV**_**min**_. (c) *γ*_**SMV**_. (d) SMA. (e) **E**. (f) *μ*_**R**_. Standard movements.

**Figure 21:** Multiple comparison test of the means of the statistical characteristics of the sporting movements in the datasets: (a) *μ*_**SMV**_. (b) *σ*_**SMV**_. (c) *μ*_*θ*_. (d) *μ*_**SMV**_(**diff**)__. (e) *μ*_**Ap**_. (f) **A**_*ω*_**diff**(**max**)__. Sporting movements.

**Figure 22:** Multiple comparison test of the means of the statistical characteristics of the sporting movements in the datasets: (a) **SMV**_**max**_. (b) **SMV**_**min**_. (c) *γ*_**SMV**_. (d) SMA. (e) **E**. (f) *μ*_**R**_. Sporting movements.

**Figure 23:** Multiple comparison test of the means of the statistical characteristics of the “near falls” in the two datasets that contain this type of movement: (a) *μ*_**SMV**_. (b) *σ*_**SMV**_. (c) *μ*_*θ*_. (d) *μ*_**SMV**_(**diff**)__. (e) *μ*_**Ap**_. (f) **A**_*ω*_**diff**(**max**)__.

**Figure 24:** Multiple comparison test of the means of the statistical characteristics of the “near falls” in the two datasets that contain this type of movement: (a) **SMV**_**max**_. (b) **SMV**_**min**_. (c) *γ*_**SMV**_. (d) SMA. (e) **E**. (f) *μ*_**R**_. Near falls.

**Figure 25:** Multiple comparison test of the means of the statistical characteristics of the movements labelled as “walking” in the seven datasets that contain this type of ADL (sensor located on the waist): (a) *μ*_**SMV**_. (b) *σ*_**SMV**_. (c) *μ*_*θ*_. (d) *μ*_**SMV**_(**diff**)__. (e) *μ*_**Ap**_. (f) **A**_*ω*_**diff**(**max**)__.

**Figure 26:** Multiple comparison test of the means of the statistical characteristics of the movements labelled as “walking” in the seven datasets that contain this type of ADL (sensor located on the waist): (a) **SMV**_**max**_. (b) **SMV**_**min**_. (c) *γ*_**SMV**_. (d) SMA. (e) **E**. (f) *μ*_**R**_.

**Figure 27:** Multiple comparison test of the means of the statistical characteristics of the datasets for the measurements on the wrist and ADL movements: (a) *μ*_**SMV**_. (b) *σ*_**SMV**_. (c) *μ*_*θ*_. (d) *μ*_**SMV**_(**diff**)__. (e) *μ*_**Ap**_. (f) **A**_*ω*_**diff**(**max**)__.

**Figure 28:** Multiple comparison test of the means of the statistical characteristics of the datasets for the measurements on the wrist and ADL movements: (a) **SMV**_**max**_. (b) **SMV**_**min**_. (c) *γ*_**SMV**_. (d) SMA. (f) **E**. (f) *μ*_**R**_.

**Figure 29:** Multiple comparison test of the means of the statistical characteristics of the datasets for the measurements on the wrist and fall movements: (a) *μ*_**SMV**_. (b) *σ*_**SMV**_. (c) *μ*_*θ*_. (d) *μ*_**SMV**_(**diff**)__. (e) *μ*_**Ap**_. (f) **A**_*ω*_**diff**(**max**)__.

**Figure 30:** Multiple comparison test of the means of the statistical characteristics of the datasets for the measurements on the wrist and ADL movements: (a) **SMV**_**max**_. (b) **SMV**_**min**_. (c) *γ*_**SMV**_. (d) SMA. (f) **E**. (f) *μ*_**R**_.

**Table 1:** Authors and references of the existing public datasets (^*∗*^the check mark indicates those datasets employed in this study).

Dataset	Ref.	Authors	Institution	City (country)	Year	^*∗*^
DLR	[29]	Frank et al.	German Aerospace Center (DLR)	Munich (Germany)	2010	√
LDPA	[30]	Kaluza et al.	Jožef Stefan Institute	Ljubljana (Slovenia)	2010	
MobiFall	[31]	Vavoulas et al.	BMI Lab (Technological Educational Institute of Crete)	Heraklion (Greece)	2013	
MobiAct	[32]				2016	
EvAAL	[33]	Kozina et al.	Department of Intelligent Systems, Jozef Stefan Institute	Ljubljana (Slovenia)	2013	
TST fall detection	[34]	Gasparrini et al.	TST Group (Università Politecnica delle Marche)	Ancona (Italy)	2014	
tFall	[35]	Medrano et al.	EduQTech (University of Zaragoza)	Teruel (Spain)	2014	
UR fall detection	[36]	Kępski et al.	Interdisciplinary Center for Computational modelling (University of Rzeszow)	Krakow (Poland)	2014	
Erciyes University	[37]	Özdemir and Barshan	Department of Electrical and Electronics Engineering (Erciyes University)	Kayseri (Turkey)	2014	√
Cogent Labs	[38]	Ojetola et al.	Labs (Coventry University)	Coventry (UK)	2015	
Gravity Project	[39]	Vilarinho et al.	SINTEF ICT	Trondheim (Norway)	2015	
Graz UT OL	[40]	Wetner et al.	Graz University of Technology	Graz (Austria)	2015	
UMAFall	[41]	Casilari et al.	Dpto. Tecnología Electrónica (University of Málaga)	Málaga (Spain)	2016	√
FARSEEING	[42]	Klenk et al.	FARSEEING Consortium (SENSACTION-AAL European Commission Project)	Five hospital or scholar centers in Germany and one university in New Zealand	2016	
SisFall	[43]	Sucerquia et al.	SISTEMIC (University of Antioquia)	Antioquia (Colombia)	2017	√
UniMiB SHAR	[44]	Micucci et al.	Department of Informatics, Systems and Communication (University of Milano)	Bicocca, Milan (Italy)	2017	
SMotion	[45]	Ahmed et al.	Department of Computer Science (University of Karachi)	Karachi (Pakistan)	2017	
IMUFD	[46]	Aziz et al.	Injury Prevention and Mobility Laboratory (Simon Fraser University)	Burnaby (BC, Canada)	2017	√
CGU-BES	[47]	Wang et al.	Chang Gung University	Taoyuan (Taiwan)	2018	
CMDFALL	[48]	Tran et al.	International Research Institute MICA (Hanoi University of Science and Technology)	Hanoi (Vietnam)	2018	
DU-MD	[49]	Saha et al.	Department of Electrical and Electronic Engineering (University of Dhaka)	Dhaka (Bangladesh)	2018	
SmartFall and Smartwatch datasets	[50]	Mauldin et al.	Department of Computer Science, Texas State University	San Marcos (TX, USA)	2018	
UP-Fall	[51]	Martínez-Villaseñor et al.	Facultad de Ingeniería (Universidad Panamericana)	Mexico City (Mexico)	2019	√
DOFDA	[52]	Cotechini et al.	Department of Information Engineering (Università Politecnica delle Marche)	Ancona (Italy)	2019	√

**Table 2:** Personal characteristics of the volunteers, typology distribution, number, and duration of the executed movements.

Dataset	Number of subjects (females/males)	Age (years)	Weight (kg)	Height (cm)	Number of types of ADLs/falls	Number of samples (ADLs/falls)	Duration of the samples (s)
DLR	19 (8/11)	[23–52]	n.i.	[160–183]	15/1	1017 (961/56)	[0.27–864.33]
LDPA	5 (n.i.)	n.i.	n.i.	n.i.	10/1	100/75	Up to 300 s
MobiFall	24 (7/17)	[22–47]	[50–103]	[160–189]	9/4	630 (342/288)	[0.27–864.33]
MobiAct	57 (15/42)	[20–47]			9/4	2526 (1879/647)	[4.89–300.01]
EvAAL	1 (n.i.)	n.i.	[50–120]	[160–193]	7/1	57 (55/2)	[0.162–30.172]
TST fall detection	11 (n.i.)	[22–39]	n.i.	[162–197]	4/4	264 (132/132)	[3.84–18.34] s
tFall	10 (3/7)	[20–42]	[54–98]	[161–184]	n.i./8	10909 (9883/1026)	6 s (all samples)
UR fall detection	6 (0/6)^3^	n.i. (over 26)	n.i.	n.i.	5/4	70 (40/30)	[2.11–13.57]
Erciyes University	17 (7/10)	[19–27]	[47–92]	[157–184]	16/20	3302(1476/1826)	[8.36–37.76]
Cogent Labs	42 (6/36)	[18–51]	[43–108]	[150–187]	8/6	1968 (1520/448)	[0.53–55.73]
Gravity Project	2 (n.i.)^4^	[26–32]	[63–80]	[170–185]	7/12	117 (45/72)	[9.00–86.00]
Graz UT OL	5 (n.i.)	n.i.	n.i.	n.i.	10/4	2460 (2240/220)	[0.18–961.23]
UMAFall	19 (8/11)	[18–68]	[50–97]	[156–193]	12/3	746 (538/208)	15 s (all samples)
FARSEEING	15 (8/7)	[56–86]	[51–101]	[148–190]	0/22	22 (0/22)	1200
SisFall	38 (19/19)	[19–75]	[41.5–102]	[149–183]	19/15	4505 (2707/1798)	[9.99–179.99] s
UniMiB SHAR	30 (24/6)	[18–60]	[50–82]	[160–190]	9/8	7013 (5314/1699)	1 s (all samples)
SMotion	120 (40/71 + 9 n.i.)	[17–79]	[35–95]	[125–186]	3/1	309 (304/5)	[0.52734–27.1875]
IMUFD	10 (n.i.)	n.i.	n.i.	n.i.	8/7	600(390/210)	[15–20.01]
CGU-BES	15 (4/11)	21.8 ± 1.8	63.0 ± 10.1 kg	167.7 ± 6.0	8/4	195 (135/60)	[11.49–16.73]
CMDFALL	50 (20/30)	[21–40]	n.i.	n.i.	12/8	1000 (600/400)	450 s^1^
DU-MD	10 (4/6)	[16–22]	[40–101]	[147–185]	8/2	3299 (2309/990)	[2.85–11.55]
Smartfall	7 (n.i.)	[21–55]	n.i.	n.i.	4/4	181 (90/91)	[0.576–16.8]
Smartwatch	7 (n.i.)	[20–35]	n.i.	n.i.	7/4	2563 (2456/107)	[1–3.776]
UP-Fall	17 (8/9)	[18–24]	[53–99]	[157–175]	6/5	559(304/255)	[9.409–59.979]
DOFDA	8 (2/6)	[22–29]	[60–94]	[173–187]	5/13	432 (120/312)	1.96–17.262

1. For the CMDFAL dataset, all the 20 programmed movements are executed in a continuous manner during 7.5 minutes. 2. n.i.: not indicated by the authors.

**Table 3:** Position and characteristics of the sensor used in the different datasets.

Dataset	Number of sensing points	Captured signals in each sensing point	Positions of the sensing points	Type of device	Sampling rate (Hz)	Range
DLR	1	3 (A, G, M)	Waist (belt)	1 external IMU	100	±5 g (A)
						±1200°/s (G)
						±75 *μ*T (M)
LDPA	4	Position (x,y,z coordinates)	Right ankle, left ankle, waist (belt), and chest	4 external IMUS (tags)	10	Tens of meters
MobiFall and MobiAct	1	3 (A, G, O)	Thigh (trouser pocket)	1 smartphone	87 (A)	±2 g (A)
					100 (G,O)	±200°/s (G)
						±360° (O)
EvAAL	2	1 (A)	Chest and right thigh	2 external IMUs	50	±16 g (A)
TST fall detection	2	1 (A)	Waist and wrist	2 external IMUs	100	±8 g (A)
Erciyes University	6	3(A, G, M)	Chest, head, ankle, thigh, wrist, and waist	6 external IMUs	25	±16 g (A)
						±1200°/s (G)
						±150 *μ*T (M)
tFall	1	1 (A)	Alternatively: thigh (right or left pocket) and hand bag (left or right side)	1 smartphone	45 (±12)	±2 g (A)
UR fall detection	1	1 (A)	Waist (near the pelvis)	1 external IMU	256	±8 g (A)
Cogent Labs	2	2 (A, G)	Chest and thigh	2 external IMUs	100	±8 g (A)
						±2000°/s (G)
Gravity Project	2	1 (A)	Thigh (smartphone in a pocket)	1 smartphone	50 (SP)	±16 g (A)
			Wrist (smartwatch)	1 smartwatch	157 (SW)	±2 g (A)
Graz UT OL	1	2 (A, O)	Waist (belt bag)	1 smartphone^3^	5	±2 g (A)
						±360° (O)
UMAFall	5	3(A, G, M)	Ankle, chest, thigh, and waist	1 smartphone^4^	100 (SP)	±16 g (A)
			Wrist	4 external IMUs	20 (IMUs)	±256°/s (G)
						±4800 *μ*T (M)
FARSEEING	1	2 (A,G)	Waist or thigh	1 external IMU	100	±6 g (A)
						±100°/s (G)
SisFall	1	3 (A, A, G)	Waist	2 accelerometers and a gyroscope in a single mode	200	±16 g (A1)
						±8 g (A2)
						±2000°/s (G)
UniMiB SHAR	1	1 (A)	Thigh (left or right trouser pocket)	1 smartphone	50	±2 g (A)
SMotion	1	A, G	Waist	1 external IMU	51	±4 g (A2)
						±500°/s (G)
IMUFD	7	3(A, G, M)	Chest, head, left ankle, left thigh, right ankle, right thigh, and waist	7 external IMUs	128	±16 g (A)
						±2000°/s (G)
						±800 *μ*T (M)
CGU-BES	1	2 (A, G)	Chest	1 sensing mote with a gyroscope and accelerometer	200	±3.6 g (A)
						±400°/s (G)
CMDFALL^1^	2	1 (A)	Left wrist and left hip	1 external IMU	50	±16 g (A)
DU-MD	1	1 (A)	Wrist	1 external IMU	33	±4 g (A)
SmartFall	1	1 (A)	Wrist	1 external IMU	31.25	±16 g (A)
Smartwatch	1	1 (A)	Wrist (left hand)	Smartwatch (MS band)	31.25	±8 g (A)
UP-Fall	5	2 (A, G)	Ankle, neck, and thigh (pocket)	5 external IMUs	14	±8 g (A)
			Waist and wrist			±2000°/s (G)
DOFDA	1	4 (A, G, O, M)	Waist	1 external IMU	33	±16 g (A)
						±2000°/s (G)
						±800 *μ*T (M)

*Note.* A : accelerometer, G : gyroscope, O : orientation measurements, M : magnetometer, SP : smartphone. 1. TST, UR, CMDFALL, and UP datasets also include the measurements (RGB, depth, and skeleton information) of Kinect sensors or video cameras, not considered in this Table 2. n.i.: not indicated by the authors.

**Table 4:** Distribution of the activities in the traces among the different considered general types of movements.

Dataset	DLR	DOFDA	Erciyes U.	IMUFD	SisFall	UMAFall	UP-fall
Number of types of ADLs/falls	15/1	5/13	16/20	8/7	19/15	12/3	6/5
BASIC MOVEMENTS	4	2	8	4	11	7	3
Standing	1			1			1
Rising/descending from(to) lying/kneeling	1	1	1	1	2	1	
Lying	1		1		1		1
Descending to sitting/rising from sitting	1	1	4	2	8	1	1
Bending			1			1	
Hand movements (making a call and applauding)						4	
Others			1				
STANDARD MOVEMENTS	4	3	5	4	4	3	2
Walking	1	1	2	1	2	1	1
Going down	1						
Climbing stairs (up and/or down)	2	1		2	2	2	
Picking		1	1	1			1
Others			2				
SPORTING MOVEMENTS	7		1		3	2	1
Running/Jogging	1		1		2	2	
Jumping/Hopping	4				1		1
Others	2						
NEAR FALLS			2		1		
Stumble			1		1		
Trip			1				
FALLS	1	13	20	7	15	3	5
Backwards		4	4		2	1	1
Forward/Frontal		4	8		2	1	2
Lateral		4	4		2	1	1
Slipping				1	3		
Tripping/hitting/bumping				2	2		
Missteps				3			
Syncope/Fainting/collapse		1	2	1	4		
Others	1		2				1

## Data Availability

Datasets employed in this paper are publicly available in the Internet. URLs to access the data are provided by their authors in the corresponding references (see References).

## References

[1] World Health Organization (WHO) (2018). Falls (facts sheet, 16 January 2018).

[2] Lord S. R., Sherrington C., Menz H. B., Close J. C. T. (2007). *Falls in Older People: Risk Factors and Strategies for Prevention*.

[3] Ku Y.-C., Liu M.-E., Tsai Y.-F., Liu W.-C., Lin S.-L., Tsai S.-J. (2013). Associated factors for falls, recurrent falls, and injurious falls in aged men living in taiwan veterans homes. *International Journal of Gerontology*.

[4] Becker C., Schwickert L. (2012). Proposal for a multiphase fall model based on real-world fall recordings with body-fixed sensors. *Zeitschrift für Gerontologie und Geriatrie*.

[5] Kangas M., Vikman I., Nyberg L., Korpelainen R., Lindblom J., Jämsä T. (2012). Comparison of real-life accidental falls in older people with experimental falls in middle-aged test subjects. *Gait Posture*.

[6] Klenk J., Becker C., Lieken F. (2011). Comparison of acceleration signals of simulated and real-world backward falls. *Medical Engineering & Physics*.

[7] Bagalà F. (2012). Evaluation of accelerometer-based fall detection algorithms on real-world falls. *PLoS One*.

[8] Aziz O. (2017). Validation of accuracy of SVM-based fall detection system using real-world fall and non-fall datasets. *PLoS One*.

[9] FARSEEING (2015). Fall repository for the design of smart and self-adaptive environments prolonging independent living project.

[10] UCI Machine Learning Repository (2020). Human activity recognition using smartphones data set.

[11] Davis K. A., Owusu E. B. (2020). Smartphone dataset for human activity recognition-dataset by uci | data.world.

[12] Anderson D., Luke R., Keller J. M., Skubic M. (2008). CIRL fall recognition resources.

[13] Charfi I., Miteran J., Dubois J., Atri M., Tourki R. (2013). Optimized spatio-temporal descriptors for real-time fall detection: comparison of support vector machine and Adaboost-based classification. *The Journal of Electronic Imaging*.

[14] Ma X., Wang H., Xue B., Zhou M., Ji B., Li Y. (2014). Depth-based human fall detection via shape features and improved extreme learning machine. *IEEE Journal of Biomedical and Health Informatics*.

[15] Zhang Z., Conly C., Athitsos V. (2014). Evaluating depth-based computer vision methods for fall detection under occlusions. *Lecture Notes in Computer Science (including subseries Lecture Notes in Artificial Intelligence and Lecture Notes in Bioinformatics)*.

[16] Riquelme F., Espinoza C., Rodenas T., Minonzio J.-G., Taramasco C. (2019). eHomeSeniors dataset: an infrared thermal sensor dataset for automatic fall detection research. *Sensors*.

[17] Auvinet E., Rougier C., Meunier J., St-Arnaud A., Rousseau J. (2010). Multiple cameras fall dataset. *DIRO-Université Montréal (Canada)*.

[18] Baldewijns G., Vanrumste B., Debard G., Croonenborghs T., Mertes G. (2016). Bridging the gap between real-life data and simulated data by providing a highly realistic fall dataset for evaluating camera-based fall detection algorithms. *Healthcare Technology Letters*.

[19] Czygan F. C., Athitsos V. (1976). “Synthetical” aiptasia mutabilis RAPP (coelenterata) (author’s transl). *Zeitschrift Fur Naturforschung*.

[20] Aslan M., Akbulut Y., Şengür A., İnce M. C. (2017). Eklem tabanlı etkili düşme tespiti. *Gazi Üniversitesi Mühendislik-Mimarlık Fakültesi Dergisi*.

[21] MEBIOMEC (Universidad Politécnica de Valencia (2020). Fall detection testing dataset.

[22] Mastorakis G., Makris D. (2014). Fall detection system using Kinect’s infrared sensor. *Journal of Real-Time Image Processing*.

[23] Adhikari K., Bouchachia H., Nait-Charif H. Activity recognition for indoor fall detection using convolutional neural network.

[24] Khojasteh S. B., Villar J. R., Chira C., González V. M., de la Cal E. (2018). Improving fall detection using an on-wrist wearable accelerometer. *Sensors*.

[25] Leutheuser H., Schuldhaus D., Eskofier B. M., Fukui Y., Togawa T. (2013). Hierarchical, multi-sensor based classification of daily life activities: comparison with state-of-the-art algorithms using a benchmark dataset. *PLoS One*.

[26] Villar J. R., Vergara P., Menéndez M., de la Cal E., González V. M., Sedano J. (2016). Generalized models for the classification of abnormal movements in daily life and its applicability to Epilepsy convulsion recognition. *International Journal of Neural Systems*.

[27] Igual R., Medrano C., Plaza I. (2015). A comparison of public datasets for acceleration-based fall detection. *Medical Engineering & Physics*.

[28] Casilari E., Lora-Rivera R., García-Lagos F. (2020). A study on the application of convolutional neural networks to fall detection evaluated with multiple public datasets. *Sensors*.

[29] Frank K., Vera Nadales M. J., Robertson P., Pfeifer T. Bayesian recognition of motion related activities with inertial sensors.

[30] Kaluža B., Mirchevska V., Dovgan E., Luštrek M. An agent-based approach to care in independent living.

[31] Vavoulas G., Pediaditis M., Spanakis E. G., Tsiknakis M. The MobiFall dataset: an initial evaluation of fall detection algorithms using smartphones.

[32] Vavoulas G., Chatzaki C., Malliotakis T., Pediaditis M. The mobiact dataset: recognition of activities of daily living using smartphones.

[33] Kozina S., Gjoreski H., Gams M., Luštrek M. (2013). Three-layer activity recognition combining domain knowledge and meta-classification. *Journal of Medical and Biological Engineering*.

[34] Gasparrini S., Cippitelli E., Spinsante S., Gambi E. (2014). A depth-based fall detection system using a Kinect sensor. *Sensors*.

[35] Medrano C., Igual R., Plaza I., Castro M. (2014). Detecting falls as novelties in acceleration patterns acquired with smartphones. *PLoS One*.

[36] Kwolek B., Kepski M. (2014). Human fall detection on embedded platform using depth maps and wireless accelerometer. *Computer Methods and Programs in Biomedicine*.

[37] Özdemir A., Barshan B. (2014). Detecting falls with wearable sensors using machine learning techniques. *Sensors*.

[38] Ojetola O., Gaura E., Brusey J. Data set for fall events and daily activities from inertial sensors.

[39] Vilarinho T. A combined smartphone and Smartwatch fall detection system.

[40] Wertner A., Czech P., Pammer-Schindler V. An open labelled dataset for mobile phone sensing based fall detection.

[41] Casilari E., Santoyo-Ramón J. A., Cano-García J. M. (2016). Analysis of a smartphone-based architecture with multiple mobility sensors for fall detection. *PLoS One*.

[42] Klenk J. (2016). The FARSEEING real-world fall repository: a large-scale collaborative database to collect and share sensor signals from real-world falls. *European Review of Aging and Physical Activity*.

[43] Sucerquia A., López J. D., Vargas-bonilla J. F. (2017). SisFall : A fall and movement dataset. *Sensors*.

[44] Micucci D., Mobilio M., Napoletano P. (2017). UniMiB SHAR: a new dataset for human activity recognition using acceleration data from smartphones. *Applied Science*.

[45] Ahmed M., Mehmood N., Nadeem A., Mehmood A., Rizwan K. (2017). Fall detection system for the elderly based on the classification of shimmer sensor prototype data. *Healthcare Informatics Research*.

[46] Aziz O., Musngi M., Park E. J., Mori G., Robinovitch S. N. (2017). A comparison of accuracy of fall detection algorithms (threshold-based vs. machine learning) using waist-mounted tri-axial accelerometer signals from a comprehensive set of falls and non-fall trials. *Medical & Biological Engineering & Computing*.

[47] Wang F. T., Chan H. L., Hsu M. H., Lin C. K., Chao P. K., Chang Y. J. (2018). Threshold-based fall detection using a hybrid of tri-axial accelerometer and gyroscope. *Physiological Measurement*.

[48] Tran T. H. A multi-modal multi-view dataset for human fall analysis and preliminary investigation on modality.

[49] Saha S. S., Rahman S., Rasna M. J., Mahfuzul Islam A. K. M., Rahman Ahad M. A. DUMD: An open-source human action dataset for ubiquitous wearable sensors.

[50] Mauldin T., Canby M., Metsis V., Ngu A., Rivera C. (2018). SmartFall: a smartwatch-based fall detection system using deep learning. *Sensors*.

[51] Martínez-Villaseñor L., Ponce H., Brieva J., Moya-Albor E., Núñez-Martínez J., Peñafort-Asturiano C. (2019). UP-fall detection dataset: a multimodal approach. *Sensors*.

[52] Cotechini V., Belli A., Palma L., Morettini M., Burattini L., Pierleoni P. (2019). A dataset for the development and optimization of fall detection algorithms based on wearable sensors. *Data BR*.

[53] Zhao G., Mei Z., Liang D. (2012). Exploration and implementation of a pre-impact fall recognition method based on an inertial body sensor network. *Sensors*.

[54] Gjoreski H., Luštrek M., Gams M. Accelerometer placement for posture recognition and fall detection.

[55] Dai J., Bai X., Yang Z., Shen Z., Xuan D. PerFallD: A pervasive fall detection system using mobile phones.

[56] Kangas M., Konttila A., Lindgren P., Winblad I., Jämsä T. (2008). Comparison of low-complexity fall detection algorithms for body attached accelerometers. *Gait & Posture*.

[57] Fang S.-H., Liang Y.-C., Chiu K.-M. Developing a mobile phone-based fall detection system on android platform.

[58] Casilari E., Álvarez-Marco M., García-Lagos F. (2020). A Study of the use of gyroscope measurements in wearable fall detection systems. *Symmetry*.

[59] Liu S.-H., Cheng W.-C. (2012). Fall detection with the support vector machine during scripted and continuous unscripted activities. *Sensors*.

[60] Santoyo-Ramón J., Casilari E., Cano-García J. (2018). Analysis of a smartphone-based architecture with multiple mobility sensors for fall detection with supervised learning. *Sensors*.

[61] Abbate S., Avvenuti M., Bonatesta F., Cola G., Corsini P., Vecchio A. (2012). A smartphone-based fall detection system. *Pervasive and Mobile Computing*.

[62] Bourke A. K., O’Donovan K. J., Nelson J., ÓLaighin G. M. Fall-detection through vertical velocity thresholding using a tri-axial accelerometer characterized using an optical motion-capture system.

[63] Karantonis D. M., Narayanan M. R., Mathie M., Lovell N. H., Celler B. G. (2006). Implementation of a real-time human movement classifier using a triaxial accelerometer for ambulatory monitoring. *IEEE Transactions on Information Technology in Biomedicine*.

[64] Ojetola O., Gaura E. I., Brusey J. Fall detection with wearable sensors--safe (smart fall detection).

[65] Putra I. P. E. S., Vesilo R. Genetic-algorithm-based feature-selection technique for fall detection using multi-placement wearable sensors.

[66] Özdemir A. T. (2016). An analysis on sensor locations of the human body for wearable fall detection devices: principles and practice. *Sensors (Switzerland)*.

[67] Vallabh P., Malekian R., Ye N., Bogatinoska D. C. Fall detection using machine learning algorithms.

[68] Wang C., Redmond S. J., Lu W., Stevens M. C., Lord S. R., Lovell N. H. (2017). Selecting power-efficient signal features for a low-power fall detector. *IEEE Transactions on Bio-Medical Engineering*.

[69] Kansiz A. O., Guvensan M. A., Turkmen H. I. Selection of time-domain features for fall detection based on supervised learning.

[70] Sucerquia A., López J. D., Vargas-Bonilla J. F. (2018). Real-life/real-time elderly fall detection with a triaxial accelerometer. *Sensors*.

[71] Chernbumroong S., Cang S., Yu H. (2015). Genetic algorithm-based classifiers fusion for multisensor activity recognition of elderly people. *IEEE Journal of Biomedical and Health Informatics*.

[72] Bersch S., Azzi D., Khusainov R., Achumba I., Ries J. (2014). Sensor data acquisition and processing parameters for human activity classification. *Sensors*.

[73] Vallabh P., Malekian R. (2018). Fall detection monitoring systems: a comprehensive review. *Journal of Ambient Intelligence and Humanized Computing*.

[74] Xi X., Tang M., Miran S. M., Luo Z. (2017). Evaluation of feature extraction and recognition for activity monitoring and fall detection based on wearable sEMG sensors. *Sensors (Switzerland)*.

[75] Chen K.-H., Yang J.-J., Jaw F.-S. (2016). Accelerometer-based fall detection using feature extraction and support vector machine algorithms. *Instrumentation Science & Technology*.

[76] Casilari E., Santoyo-Ramón J. A., Cano-García J. M. (2017). Analysis of public datasets for wearable fall detection systems. *Sensors*.

